The article "Application of Digital Information Technology in Book Classification and Quick Search in University Libraries" was retracted in 2023. Reasons: unreliable results or conclusions; concerns about the data; concerns about the results or conclusions; concerns about the peer review.

# Application of Digital Information Technology in Book Classification and Quick Search in University Libraries

**DOI:** 10.1155/2022/4543467

**Published:** 2022-08-05

**Authors:** Huijie Xiao

**Affiliations:** Wenzhou Vocational College of Science and Technology, Wenzhou 325006, Zhejiang, China

## Abstract

A digital library is a digital information resource system supported by modern high technology, a next-generation information resource management model on the Internet, and the result of the digitization of library collections, and with the development of society and the accelerated pace of people's lives, people cannot spend too much time classifying and finding books, so the study of book classification and quick finding in university libraries is very important. This paper mainly researches and analyzes the classification and quick search of books in the university library through the algorithms and methods of digital information technology and finds a better algorithm. This paper mainly conducts experiments on automatic text and support vector machine (one-to-many and global optimization) methods and compares the obtained experimental data, such as classification accuracy, classification time, search time, and other data. The experimental results show that the classification accuracy of these three classification methods is in the range of 86%–94%. However, compared with the two methods of automatic text classification and one-to-many classification, the global optimization classification has the highest accuracy in the sample size of each interval. Among them, the classification time is the lowest for automatic text classification, which is less than 30s, and the one-to-many classification sample takes the most time, and their average fitness is in the range of 24%–27%.

## 1. Introduction

With the rapid development of computer and Internet technology, many fields of human society have been affected, and even great changes have taken place. Therefore, the digital library is also produced in the digital age, and the digital library is no longer limited to the traditional library. Building a book industry requires a new way of thinking, which involves not only the transition from traditional libraries to digital libraries but also the mature and pioneering research and practice of creating next-generation digital libraries on the Internet. But, now there is not much research on the digital library. They focus on the human-computer interaction aspect of the study, but ignore the most important aspect of the digital library, book classification, and fast search. A good algorithm can greatly reduce the time in book classification and fast search. It is therefore very important to find a better algorithm and apply it to the digital library, which has become the research direction of researchers nowadays.

Because a digital library is a new field of computer application, including many technologies such as the Internet, multimedia, data storage, data mining, and intellectual property protection, its application and trade prospects are very broad, which is in line with the current digital information age, and a digital library can greatly improve people's learning efficiency. It is important to reduce the time it takes for people to find books and for librarians to sort books. Then, the research on book classification and quick search is of great significance.

This paper mainly analyzes the working principle of automatic text classification and support vector machine and then makes a corresponding system based on these two classification methods. We use the real data collection of the Sogou News Chinese Text Classification corpus on Sogou Lab as the experimental sample. There are a total of 2000 text data samples; we also start the experiment, record the data, and analyze the advantages and disadvantages of the method.

The innovation of this paper is as follows: (1) this paper introduces the automatic text classification method and various algorithms in it, as well as various methods and principles in support vector machines. (2) This paper compares the three methods of automatic text, one-to-many, and global optimization, and then summarizes their advantages and disadvantages. (3) This paper also provides a specific introduction to the theory, functions, and components of human-computer interaction and also introduces some optimization issues for interactive user interfaces.

## 2. Related Work

At present, more and more researchers have studied the classification and quick search of books in the digital library. Among them, Li S studied the modern big data information technology, content, and relationship through the case analysis of China Digital Library and found that the blockchain can achieve more accurate information collection, safer information storage, and more effective information dissemination. On this basis, we construct a relatively complete application scenario of modern information technology in the digital library [1]. Paletta examined information technology life cycle management to support digital libraries and examined the dynamics of information technology and its ability to generate innovations that directly affect the quality of digital library services. Use these new technologies to help improve the quality of services provided by digital libraries [2]. But, there is no large-scale experimental verification. Sonkar, in order to distinguish between relevant and nonrelevant information, studies all issues related to the development of the digital library of clippings, dealing with various open issues that arise in the field, addressing challenges such as metadata selection, preservation, technical obsolescence, and copyright issues [3]. Yadav studied the classification and preservation techniques of traditional documents and digital resources used by selected libraries in New Delhi, India, and solved the difficult task for libraries to access these resources in the future [4]. But, the cost is too high. Kato's research considers the development, awareness, adoption, and use of digital library (DL) resources at the university level. He uses these important properties of DL services to reveal the simplicity of online information access and the performance of DL utilities [5]. Linlin studied the application of information processing technology in university libraries in the era of big data. 2D virtual environments based on text and images are gradually transforming into more and more realistic and detailed 3D virtual environments. He proposed a three-step strategy for developing a virtual library: preparation, pilot modeling, and application [6]. Umeozor investigated the evaluation of image reuse in digital libraries for applications of content-based image retrieval (CBIR) and reverse image lookup (RIL). It also briefly analyzed 4 published case studies of image reuse assessment in digital libraries [7]. But, the comparison of other methods is lacking.

## 3. Theoretical Knowledge and Methods

### 3.1. Digital Libraries

The development of computers, networks, and communications has greatly improved the ability to generate, process, and disseminate digital information [8]. Digital information is easier to store, transmit, and process than other forms of stored information [9]. Digital information resources need system technology because traditional information management methods, such as library management and audio-visual file management, can no longer adapt to the development of modern social technology. Many problems in the field of computer and Internet technology have not been fully solved. How to organize, extract, acquire, and intelligently and efficiently utilize all kinds of massive digital information, and how to effectively utilize the advantages of the “Internet” are the first problems to be solved at present [10]. In response to these problems, scientists put forward the concept of the digital library. Its basic architecture diagram is shown in Figure 1.

A digital library is a digital information material system supported by modern technology, and it is the next-generation information resource management model of China's Internet. The digital library is an important achievement of the comprehensive digitization of Chinese library collections [11, 12], and the university library refers to the library that serves the teaching and scientific research of higher education, and is the document and information center of higher education. With the rapid development of science and technology, traditional libraries cannot meet the current needs of people's learning, and are developing in the direction of digital libraries. At present, most of the documents in the library are electronic books, periodicals, electronic newspapers, and research reports. They can also link to existing digital resource websites through the Internet so that the materials that need to be managed are not only the library's documents but also some other websites. In this way, the research scope of digital library goes far beyond the field of conventional library. It is already a digital information technology with diversified media and colorful information [13], and compared with other models of libraries, digital libraries have many advantages as shown in Table 1.

### 3.2. Automatic Text Classification Methods

A digital library is a powerful knowledge base. The digital library service center is mainly for people, not books. The characteristics of the data library deepen its business to the information level, and through the intelligent combination and management of information, the resources are established as an information system [14].

Text classification is the process of assigning large amounts of text into one or more categories based on the content or properties of the text. A text classification algorithm is a supervised learning algorithm. It should include a set of manually classified training materials and specific document categories. Based on this trained model, we create a classifier and then classify new documents. Therefore, existing data processing methods cannot be directly applied. We must preprocess the text, extracting metadata representing its attributes. Metadata, also known as intermediate data and relay data, mainly describe the information of data attributes, and have functions such as indicating storage location, historical data, resource search, and file recording. Metadata is considered an electronic type of catalogue, in order to achieve the purpose of cataloguing. For hard-to-represent entities, the first step is to find a computer-processable representation, the target representation. The process of creating a target representation is the process of creating a mining model [15]. For Chinese, documents must also be tokenized beforehand. There are many types of target representation models. Boolean type, vector space type, and probability type, etc., are commonly used. The Boolean model means simply stating whether a feature is present in a document using 0 and 1, with 0 indicating absence and 1 indicating presence. This representation has the advantage of simplicity, but does not convey the relative importance of information about different features very well and is rarely used in practice. The probabilistic model counts the probability that the document to be classified is in each category and thus selects the most likely category tokens. The disadvantage of this model is that it does not take into account the frequency of index terms within the text. In recent years, vector space modeling methods are the most widely used and effective object representation methods.

Feature extraction plays a key role in text analysis; it helps to reduce the dimension of the vector space and simplify the algorithm, thus avoiding overfitting [16]. Because of the exponential correlation between the number of feature subsets and the number of features, it is almost impossible to enumerate features, so one assumes that features are independent of each other. Therefore, the feature extraction method is modified by the feature subset extraction method. Through the scoring function of each specific feature, the score of each feature and the division method of each digital library feature can be counted and then arranged according to the score, and thousands of words with the largest score are selected as feature words. The method of feature extraction in text classification is based on the Gini coefficient. The Gini coefficient is a concept in economics that takes on a value between 0 and 1. A value of 0 indicates a very even distribution of income, a value of 1 indicates that the income of a country is in the hands of a certain person, a value within a certain range indicates a reasonable distribution, a value below (usually) 0.2 indicates a lack of power, and a value above (usually) 0.4 indicates an unreasonable distribution.

In the vector space model, a certain weight *W* is assigned according to its importance in the document. We can think of it as an *n*-dimensional coordinate system; *W*_1_, *W*_2_,…, *W*_*n*_ is the corresponding coordinate value. Therefore, each document can be mapped to a point in a vector space consisting of a set of word vectors, and all user targets or unknown documents can be represented by word feature vectors. Thus, the document information classification problem is transformed into a vector space to solve the vector matching problem. Suppose the user's target is *U* and the unknown document is *V*, then the similarity between them can be measured by the angle between the vectors. The smaller the angle, the greater the similarity. The similarity calculation formula is as follows:

(1) $$\begin{array}{c} \text{Sim}m\left(V,U\right)=\cos\left(V,U\right). \end{array}$$

The main advantage of the vector space model is its huge advantage in knowledge representation methods. In this model, the formalization of text content as a point in multidimensional space is given to a vector, which greatly reduces the complexity of the problem, reducing the processing of text content to vector operations in vector space [17]. The calculation of weights can be done manually with rules or automatically with statistics, which makes it easy to combine the advantages of statistical and rule methods. Defining the text in the real number domain as a vector, many established calculation methods in pattern recognition and other fields can be applied, which greatly improves the computability and operability of natural language text. Therefore, the formal method of text representation, the vector space model, is the basis and prerequisite for realizing various text processing applications.

There are three main categories of text classification algorithms that are commonly used. The basic idea is to use the TFIDF weight formula to calculate the importance of a word in a document and then use the cosine distance to calculate the similarity of two word vectors, which includes the TFDF algorithm, and the k-nearest neighbor algorithm. Another class of methods is based on probability and information theory classifiers, such as pure Bayesian. Another class of methods is based on probability and information theory, such as pure Bayesian algorithm and maximum entropy algorithm; the third class is based on knowledge learning methods, such as decision tree and other algorithms.

The simple way of dividing the distance between text vectors is that each text category first generates a center vector representing the category, which is determined by the arithmetic mean. Then, we define a new text vector when new text appears and determine the distance (similarity) between the vector and the center vector to calculate each category and finally determine what type of new text is most similar to the given text. The formula is

(2) $$\begin{array}{c} \text{Sim}m\left(d_{i},d_{j}\right)=\frac{\sum_{k=1}^{M}W_{ik}\times W_{jk}}{\sqrt{\left(\sum_{k=i}^{M}W_{ik}^{2}\right)\left(\sum_{k=i}^{M}W_{jk}^{2}\right)}}. \end{array}$$

Among them, *d*_*i*_ is the feature vector of the new text, *d*_*j*_ is the center vector of the *j*-th class, *M* is the dimension of the feature vector, and *W*_*k*_ is the *K*th dimension of the vector.

The nearest neighbor method is one of the most important nonparametric methods in pattern recognition. The idea of the KNN algorithm is very simple: given an object to be recognized, the system finds the *k*-nearest neighbors in the learning set, sees which category the *k*-nearest neighbors belong to, and assigns the sample to the category to be recognized. The nearest neighbor classifier extracts the element that is most similar to the element to be identified from the classified elements, thereby obtaining the category of the detected element [18].

There are two definitions for the statistical word in the file, one is the binomial assignment, that is, if the word appears in the file, it is assigned a value of 1; otherwise, it is assigned a value of 0, so the calculation is relatively simple. The other is to count the frequency of words appearing in the document, which allows the algorithm to use more information and achieve a higher classification accuracy than the first definition. After calculating the word frequency matrix, weights are assigned to the vectors in the document according to the formula TFIDF [19, 20].

(3) $$\begin{array}{c} W_{ik}=tf_{ik}*i\;df_{k},\\ idf_{k}=\log\left(N/df_{k}+1\right), \end{array}$$

where *N* is the number of documents, *tf*_*ik*_ refers to the frequency of the *k*-th word in the *i*-th document, and *df*_*k*_ refers to the number of documents that contain the *k*-th word in the entire training set. The distance formula is

(4) $$\begin{array}{c} \cos\left({\overset{⟶}{d}}_{i},{\overset{⟶}{d}}_{j}\right)=\frac{{\overset{⟶}{\text{d}}}_{i}•{\overset{⟶}{\text{d}}}_{j}}{\left\|{\overset{⟶}{\text{d}}}_{i}\right\|•\left\|{\overset{⟶}{\text{d}}}_{j}\right\|}, \end{array}$$

where *d*_*i*_ is the feature vector of the new text and *d*_*j*_ is the centroid vector of class *j*. It is mainly a dot product calculation.

A Bayesian probabilistic classifier treats an article as a set of independent words. From the training set, we determine the probability that each word belongs to a different class according to Bayesian theory and build a Bayesian model. The basic idea of the algorithm is to calculate the probability that a text fragment belongs to a certain category, and the probability that a text fragment belongs to a certain category is equal to the exhaustive formula of the probability that each word in the text belongs to this category. This classification algorithm must compute as follows:

(1) Calculate the probability vector (*w*_1_, *w*_2_,…, *w*_*n*_) of the feature word belonging to each category:
  (5) $$\begin{array}{c} w_{k}=P\left(W_{k}|C_{j}\right)=\frac{1+\sum_{i=1}^{\left|D\right|}N\left(W_{k},{\text{d}}_{i}\right)}{\left|V\right|+\sum_{s=1}^{\left|V\right|}\sum_{i=1}^{\left|D\right|}N\left(W_{s},{\text{d}}_{i}\right)}. \end{array}$$
(2) When a new text arrives, the words are segmented according to the feature words, and then the probability that *d*_*i*_ texts belong to *C*_*j*_ categories is calculated according to the following formula:
  (6) $$\begin{array}{c} P\left(C_{j}|d_{i};\overset{\Lambda }{\theta }\right)=\frac{P\left(C_{j}|{\text{d}}_{i}\right)\prod_{k=1}^{n}P}{\sum_{r=1}^{\left|C\right|}P\left(C_{r}|\overset{\Lambda }{\theta }\right)\prod_{k=1}^{n}P}. \end{array}$$

Among them, $P\left(C_{r}|\overset{\Lambda }{\theta }\right)$ is the similar meaning, |*C*| is the total number of classes, *N*(*W*_*k*_, *d*_*i*_) is the word frequency of *W*_*k*_ in *d*_*i*_, and *n* is the total number of feature words.

### 3.3. SVM Support Vector Machine Classification Method

Support vector machine is the most practical content in the statistical learning theory, and its theory originates from the support vector method proposed by Vapnik to solve the problem of pattern recognition [21]. SVM is a systematic approach with reproducible results. Training an SVM is quite a process of optimizing a quadratic objective function on a convex set, which does not suffer from local optima errors. SVM is a very suitable method in the field of data mining, especially for binary classification problems, especially text classification applications. Its basic idea is shown in Figure 2.

H is the error-free classification line, and *H*1 and *H*2 are lines through the closest point in each class and are parallel to the classification line. The distance between *H*1 and *H*2 is called the classification gap or classification interval between the two classes. The best classification line is one that not only separates the two sample classes without error but also maximizes the classification gap between the two sample classes. According to the principle of structural risk minimization, the first line should guarantee the minimization of empirical risk, while the second line should maximize the classification interval under the premise of minimizing the true risk, which is essentially minimizing the confidence interval of the generalized estimate [22]. In a multivariate space, the optimal classification line becomes the surface of the optimal classification. A support vector machine is a binary classification algorithm in which a set of linearly separable samples and their classes are represented as follows:

(7) $$\begin{array}{c} \left(\overset{⟶}{x_{1}},y_{1}\right),\ldots ,\left(\overset{⟶}{x_{k}},y_{k}\right)\in R^{n}\times \left\{\pm 1\right\}. \end{array}$$

The general form of the function in n-dimensional space is

(8) $$\begin{array}{c} g\left(\overset{⟶}{x}\right)=\overset{⟶}{w}•\overset{⟶}{x}+b. \end{array}$$

The classification formula is

(9) $$\begin{array}{c} \overset{⟶}{w}•\overset{⟶}{x}+b=0. \end{array}$$

Constraints should be satisfied if the classification faces all samples correctly:

(10) $$\begin{array}{c} y_{i}\left[\overset{⟶}{w}•\overset{⟶}{x}+b\right]-1\geq 0,\;i=1,2,\ldots ,k. \end{array}$$

In fact, we do not need to know the exact form of the nonlinear transformation, only its dot product operation, which we call the inner product function, also known as the kernel function [23, 24]. According to the Hilbert-Schmidt principle, if the operation satisfies the Mercer condition, then it can be used here as a dot product. Commonly used kernel functions are polynomial function, radial basis function, and sigmoid function.

(11) $$\begin{array}{c} k\left(\overset{⟶}{x_{i}},\overset{⟶}{x}\right)={\left[\left(\overset{⟶}{x_{i}},\overset{⟶}{x}\right)+1\right]}^{q},\\ k\left(\overset{⟶}{x_{i}},\overset{⟶}{x}\right)=\exp\left[-\frac{\left|\overset{⟶}{x_{i}}-\overset{⟶}{x}\right|}{\sigma^{2}}\right],\\ k\left(\overset{⟶}{x_{i}},\overset{⟶}{x}\right)=\tanh\left[v\left(\left(\overset{⟶}{x_{i}},\overset{⟶}{x}\right)+c\right)\right]. \end{array}$$

This paper mainly introduces several types of support vector machines, one-to-one and one-to-many methods, directed acyclic graph support vector machines, and global optimization classification. The one-to-one method constructs a classification surface between each class, so for *k*-class problems, *k*((*k* − 1)/2) classification functions need to be constructed. In order to distinguish the *i*-th and *j*-th samples, the following optimization problem needs to be solved:

(12) $$\begin{array}{c} \min\frac{1}{2}\left\|w^{ij}\right\|+C\sum_{j}\xi_{j}^{ij},\\ \left(w^{ij}•x\right)+b^{ij}\geq 1-\xi_{j}^{ij}. \end{array}$$

The corresponding classification function is

(13) $$\begin{array}{c} \text{sign}\left(\left(w^{ij}•x\right)+b^{ij}\right). \end{array}$$

For *k*-class problems, this method must build *k* classifiers. Among them, the *i*-th classifier treats the training samples of the *i*-th class as one class and all other classes as the other.

The directed acyclic graph algorithm is similar to one-to-one voting in the training phase, and a classification surface is also established between every two classes. However, in the classification phase, the method uses a bidirectional directed acyclic graph: *k*(*k* − 1)/2 nodes and *k* “leaves.” Each node is a binary SVM classifier and is associated with two nodes (or leaves) at the next level. When classifying unknown samples, first start from the root node of the top layer, use the classifier of the left node or right node of the next layer, and continue to classify from the root node according to the result of the classifier until it reaches a specific leaf at the bottom layer [25]. The class represented is the unknown sample class. The schematic figure of its principle is shown in Figure 3.

Global optimization classification is different from the two classification methods mentioned above. This method extends the original support vector classification method to multiclass cases and establishes a decision function to classify unknown samples at the same time. In terms of accuracy, the results obtained by this method can be compared with the one-to-many method. But, this optimization problem has to deal with all support vectors at the same time, Whereas, in other methods, the number of support vectors for the two-class independent classification problem is much smaller and the training time is proportionally less. This method can be used for many types of problems.

## 4. Application Experiment of Digital Information Technology in University Library Book Classification and Quick Search

### 4.1. Quick Search of Digital Library Based on Human-Computer Interaction

Human-computer interaction is a technology that utilizes computer input and output devices to conduct an effective dialogue between humans and computers [26]. It includes that machines provide a large amount of relevant information and request instructions through output or display devices, and humans input relevant information and requests to machines through input devices. As an independent and important research field, interactive interfaces have attracted the attention of computer manufacturers all over the world and have become another field of competition in the computer industry. As a part of the development process of computer technology, human-computer interaction technology also determines the corresponding software and hardware [27]. The development of this technology is the key to the success of a new generation of computer systems. At present, human-computer interaction is developing towards natural and harmonious human-computer interaction and user interface technology. The advancement of computer technology and the increasing amount of information in various fields of life show that the human-machine interface will become the information interface of the future. In fact, this is not only a problem of digital libraries but also of any system. Therefore, converting information to be presented on a computer using all possible techniques is a very difficult task.

The human-computer interface is an integral part of the digital library, and it is the channel for users to interact with the system when locating, searching, and retrieving information in the digital library. The person uses a simple interface to enter the keywords for the material they need, and then the digital library will look it up in the background and return the material found on the interface, which enables human-computer interaction. We make the interface completely invisible to the user. The user will be more actively looking for information and will not be bored with the work in progress. When designing an interactive user interface, people should pay attention to the following aspects: it is user-friendly, intuitive, simple, humanized, and intellectualized, making full use of images and language to enable users to understand. Grab the user's attention and provide the easiest way to use it. In a sense, the combination of virtual reality technology and information visualization will be the next generation of human-machine interface. Compared with any previous human-computer interaction technology, virtual reality technology has the greatest potential in realizing “people-oriented” and more harmonious human-machine interface. Its model is shown in Figure 4.

A lookup is the process of finding the data element with the same keyword as a given one in a number of data elements by a certain method called a lookup. It is also the process of identifying a record or data element in a lookup table with a keyword equal to the given value, based on a given value.

### 4.2. Application Experiment and Book Classification and Quick Search in University Library

This experiment uses the real data of the Sogou News Chinese text classification corpus on Sogou Lab to collect. The Chinese text classification corpus is mainly collected from a large number of real news articles saved by news portals such as Sohu. In order to ensure accurate classification, this article only selects the excerpts of the news, and it has manually grouped this part of the data, and it has all been labeled with classification. Its classification system contains seventeen category labels, which are mainly determined according to the topic of the report. It mainly includes macroeconomic reports, sports news, and technology industry reports. This paper uses some of the data as a sample for testing. The sample dataset contains 10 categories with a total of 2000 text data samples. We use 2000 of these as training samples r, each category containing approximately 200 training samples, and use 1000 of these as test samples *T*, each category containing approximately 100 test samples.

This experiment is to compare the classification accuracy of various classification methods under different sample size data, and the evaluation criteria are defined as follows:

(14) $$\begin{array}{c} \text{precision}=\frac{n_{1}}{n_{2}},\\ \text{time}=t_{1}+t_{2}, \end{array}$$

where *n*_1_ is the number of samples, *n*_2_ is the total number of samples, *t*_1_ is the training time, and *t*_2_ is the decision time. Tables 2, 3, and 4 show the approximate accuracy, time, and fitness of automatic text classification methods, one-to-many methods, and global optimization classification methods in various sample sizes.

It integrates the prepared digital library with the corresponding method and then starts the experiment. It enters the corresponding experimental samples into the digital library. It allows the system to automatically classify, and the classified data are output through the background. The experimental results are shown in Figures 5, 6, and 7:

It can be seen from the figures that the accuracy of these three classification methods is in the range of 86%–94%, but the accuracy of global optimization classification in each sample size is higher than that of automatic text classification and one-to-many classification methods. However, the classification time is the lowest in automatic text classification, all below 30s. The more the one-to-many classification samples, the more the time it takes, and their average fitness is in the range of 24%–27%. In general, automatic text classification and global optimization classification have their own advantages and disadvantages in classification, and one-to-many classification is not so good.

In order to test the stability of the automatic text classification and the global optimization classification, this paper has done many repeated experiments. The experimental data are shown in Figures 8, 9, and 10.

From the above comparison chart, we can see that the fluctuation of accuracy and fitness is relatively large, but the time is relatively stable, almost on the same line. Its description method needs further research to improve the stability of its accuracy.

After the experiment is classified, it is time to search for the data classified by the experiment. The search data are shown in Figure 11.

It can be seen from the figure that the search time increases with the increase of the sample size, but when the sample size increases to a large extent, the search time is not much different.

Comprehensive experimental data show that the accuracy of all three classification methods is in the range of 86%–94%, but automatic text classification and global optimization classification methods are more practical in classification than one-to-many classification methods, both in classification accuracy and classification time. The search time of another digital library is proportional to the sample size to a certain extent.

## 5. Discussion

This paper is mainly based on these two classification methods, namely, automatic text classification and support vector machine. This paper then makes the corresponding system based on these two methods. It then uses the real data collection of the Sogou News Chinese Text Classification corpus on Sogou Labs as experimental samples. The sample dataset contains 8 categories with a total of 2000 text data samples. It then begins sorting and finding experiments, recording data, and analyzing the strengths and weaknesses of the method. However, there are still some errors in this experiment, because it is impossible for a university library to have only 2000 books, and some will have more than tens of thousands of books. This is very different from the total sample of the experiment, and there will be dozens of categories of books. In addition, this experiment did not optimize the corresponding method, which did not improve the system accuracy on the original basis. It also does not conduct further research on the search algorithm. But, in general, the experimental data of this experiment have certain reliability. It can be used as comparative data for further optimization experiments.

## 6. Conclusion

This paper mainly compares automatic text classification, one-to-many classification, and global optimization classification. The experimental results show that the accuracy of these three classification methods is in the range of 86%–94%. However, compared with the two methods of automatic text classification and one-to-many classification, the global optimization classification has the highest accuracy in the sample size of each interval. Among them, the classification time is the lowest in automatic text classification, all below 30s. One-to-many classification samples take the most time, and their average fitness is in the range of 24%–27%. In general, automatic text classification and global optimization classification may be more suitable for application to digital libraries. Moreover, the digital libraries of these two methods are also fast in finding materials, both within 5s. The overall content shows that digital information technology will be applied to various fields in the further future research. Especially when it is applied to the classification and search of digital library, the precision and search time will be further optimized.

## Figures and Tables

**Figure 1:** Basic architecture diagram of digital library.

**Figure 2:** Basic idea of SVM.

**Figure 3:** Schematic diagram of the directed acyclic graph algorithm.

**Figure 4:** Human-computer interaction model of digital library.

**Figure 5:** Classification accuracy comparison.

**Figure 6:** Classification time comparison.

**Figure 7:** Average fitness comparison.

**Figure 8:** Accuracy comparison of multiple experiments.

**Figure 9:** Time comparison of multiple experiments.

**Figure 10:** Comparison of fitness for multiple experiments.

**Figure 11:** Lookup time comparison.

**Table 1:** Comparison of traditional and digital libraries.

	Traditional library	Digital library
Work center	Collection	User
Collection form	Printing type	Digital information resources
Way of working	Manual work	Automated processing
Retrieval means	Manual retrieval of cards	Intelligent search
Service object	Serving readers	Providing online services to global readers

**Table 2:** Approximate classification accuracy.

	0–400	400–800	800–1200	1200–1600	1600–2000
Auto text	0.87	0.88	0.9	0.92	0.93
One-to-many	0.87	0.88	0.9	0.92	0.94
Global optimization	0.88	0.89	0.92	0.93	0.94

**Table 3:** Approximate time interval.

	0–400	400–800	800–1200	1200–1600	1600–2000
Auto text	6–11	11–16	16–19	19–23	23–29
One-to-many	14–23	23–38	38–44	44–55	55–70
Global optimization	010–21	21–28	28–34	34–42	42–46

**Table 4:** Rough average fitness intervals.

	0–800	800–1500	1500–2000
Auto text	24–24.6	24–25	25–25.5
One-to-many	25.5–26	26–27	25–26
Global optimization	25–26	25.5–26	25.5–26.5

## Data Availability

No data were used to support this study.
